# Explore athletes’ sports attitude and its influence on mental health

**DOI:** 10.1016/j.heliyon.2024.e30734

**Published:** 2024-05-03

**Authors:** Xin Chen

**Affiliations:** Party School of Changzhou Wujin District Committee of the Communist Party of China, 213000, Changzhou, China

**Keywords:** Sports attitude, Athletes, Mental health, Longitudinal analysis, Correlation analysis, Regression analysis

## Abstract

This study is devoted to exploring how athletes' sports attitude affects their mental health, and explores this complex relationship through descriptive statistics, longitudinal analysis, correlation analysis and regression analysis. The research sample includes athlete data at multiple time points, covering mental health indicators such as positive attitude, negative attitude, anxiety, depression and self-esteem. Descriptive statistical results reveal the overall trend of athletes in positive attitude, anxiety, depression and self-esteem. On average, athletes show a positive attitude towards sports, but there are some variability in mental health indicators. The results of longitudinal analysis show that with the progress of the season, the positive attitude shows an upward trend, while the level of anxiety and depression shows a downward trend in some cases, which provides a detailed observation for the long-term evolution of athletes' psychological state. Correlation analysis reveals the positive correlation between positive attitude and self-esteem, positive correlation between negative attitude and anxiety, and negative correlation between teamwork attitude and depression. Regression analysis further verified the influence of positive attitude and negative attitude on anxiety. The results emphasize that the improvement of positive attitude may help to slow down the increase of anxiety level, while the increase of negative attitude may be related to the increase of anxiety. Generally speaking, the findings of this study highlight the complex relationship between athletes' mental health and their attitude towards sports. This study provides profound insights for formulating targeted psychological support strategies and emphasizes the importance of comprehensively considering multi-dimensional factors in athletes' mental health management.

## 1 Introduction

Exercise has been proved to have a positive impact on the overall health of individuals. Recent research shows that [1,2], athletes' attitude towards sports plays a vital role in shaping their mental health. These attitudes include their attitudes towards competition, their reactions to success and failure, and their views on body image and self-worth. Psychologists and sports scientists have been studying this relationship for a long time and found that a positive attitude towards sports is related to better mental health, including lower anxiety, higher self-esteem and better adaptability [3,4]. On the contrary, a negative attitude will lead to an increase in the susceptibility to depression and anxiety [5]. In addition, the mental health of athletes affects their performance in competitive sports; Those who have a positive attitude tend to remain calm under pressure and show greater adaptability and resilience. The purpose of this study is to deeply explore the complicated relationship between athletes' attitude towards sports and their mental health, and to provide more effective psychological support and training to enhance their all-round development in sports and life.

## 2 Related work

### 2.1 Athletes' attitude towards sports

Athletes' sports attitude is one of the important factors that affect their training, competitive performance and long-term career development. Athletes' psychological quality plays a vital role in their sports career, and sports attitude, as a part of psychological quality, is directly related to athletes' attitude, motivation and final performance in training and competition. In the existing research [[6], [7], [8]], there are some disputes about the definition of athletes' sports attitude and the choice of measurement tools.

The definition of athletes' attitude towards sports includes attitudes towards sports, values and beliefs related to sports. Early research mainly defined sports attitude as positive or negative emotional experience of sports activities [9,10]. With the deepening of research, the definition of sports attitude has gradually expanded to the attitude towards training, competition and teamwork, forming a more comprehensive concept.

According to the existing literature [11,12], the attitude of athletes can be decomposed into several dimensions, including but not limited to the following aspects: attitude towards training, attitude towards competition, attitude towards teamwork, trust in coaches, tolerance for failure, etc. Different dimensions of sports attitude may have different effects on athletes' performance at different stages, so in-depth study of these dimensions will help to better understand athletes' psychological state.

In order to evaluate athletes' attitude towards sports, researchers have developed various psychological measurement tools. Common tools include but are not limited to questionnaires, interviews and psychological tests [[13], [14], [15]]. Different measuring tools have different advantages and disadvantages, so researchers need to choose the appropriate tools according to the research purpose and the characteristics of the object to ensure the validity and reliability of the measurement results.

However, there are still some limitations in the current research, such as the lack of sample selection and the limitations of measurement tools. Future research can further explore the influence of different cultures and sports on athletes' attitude, and how to improve athletes' positive attitude through psychological intervention to provide more effective support for athletes' all-round development.

### 2.2 Relationship between mental health and sports attitude

Exercise is regarded as an effective way to maintain mental health, and exercise attitude is one of the important factors affecting individual sports participation and sustainability. The relationship between mental health and sports attitude has always been one of the hot spots in psychology, sports science and other fields. Exercise is not only beneficial to physical health, but also has a positive impact on mental health. Sports attitude is an important psychological factor that determines whether individuals are willing to participate in sports and continue to participate.

Research shows that [16], individuals who hold a positive attitude towards exercise are more likely to enjoy the mental health benefits brought by exercise. Positive sports attitude includes optimistic view of sports, positive recognition of physical activities and positive expectation of sports goals. These positive attitudes help to improve individual self-esteem, self-confidence, reduce the level of anxiety and depression, and promote the overall development of mental health. On the contrary, negative sports attitude may lead to the decrease of sports participation and even lead to mental health problems [17]. Negative attitudes such as negative views on sports, underestimation of one's own sports ability and pessimistic expectations of sports goals may become the trigger factors of mental health problems, including but not limited to stress, anxiety and depression.

Some studies also show that [18,19], through psychological intervention measures can effectively improve the individual's attitude towards sports, thus improving the level of mental health. Psychological education, cognitive behavioral therapy and other methods have shown certain results in changing negative attitude towards sports, which provides practical reference for sports as a means to promote mental health.

By summarizing the existing studies, we can draw the conclusion that there is a positive relationship between positive attitude towards sports and mental health. However, it is still necessary to further study the influence mechanism of sports attitude on mental health in different groups and cultural backgrounds, and how to promote positive sports attitude more effectively through psychological intervention, so as to improve the level of mental health. This has practical guiding significance for formulating mental health promotion strategies and promoting the application of sports participation in mental health treatment.

## 3 Research design and methods

### 3.1 Research sample

In this study, the athletes selected as the research object are professional football players. This choice is based on the following reasons:

Highly competitive environment. Football is a global competitive sport, and its professional level competition is highly competitive. This competitive environment may have a more significant impact on athletes' attitude towards sports, including their attitudes towards success and failure, and their views on teamwork.

Managing stress and challenges. Professional football players often face expectations from fans, the media and themselves in the game. This persistent psychological pressure and challenge may make his attitude towards sports more complicated and have a deeper impact on mental health.

Team motivation and cooperation. Football is a team sport, and the cooperation and tacit understanding between players are very important to the overall performance of the team. By studying football players, we can deeply understand how sports attitude plays a role in team motivation and cooperation, and then affect the mental health of the whole team.

In order to ensure the applicability and practicability of the study, this study selected athletes who participated in domestic or international professional football leagues to ensure the football level and competitive level of the sample [20]. In this study, the age range of the research samples is limited to 22–35 years old, so as to ensure that athletes are in the critical period of their careers and reduce the influence of age factors on the research results. Only athletes who voluntarily participate in the research are selected to ensure the ethics of the research and the reliability of the data.

It is planned to include at least 200 football players as research samples to ensure the statistical significance of the study and the representativeness of the results. At the same time, ensure that the sample includes athletes from different countries, cultures and professional leagues, so as to increase the external effectiveness and popularization of the research.

Table 1 clearly presents the elements and related descriptions of the research sample design.

**Table 1:** Elements and related descriptions of research sample design.

Sample design elements	describe
research objects	Professional football player
Sample selection reason	Global competitive sports and professional level competitions are highly competitive Facing the continuous psychological pressure from fans, media and their own expectations Football is a team sport, and the role of sports attitude in the team is explored
Sample selection criteria	Participate in domestic or international professional football leagues The age range is 22–35 years old, which is a critical period of career Only athletes who volunteered to participate in the study were selected
Sample size	At least 200 football players Athletes from different countries, cultures and professional leagues

By choosing professional football players as a specific group, we hope to understand more comprehensively how sports attitude affects mental health in a highly competitive environment and provide an empirical basis for formulating targeted psychological support and training.

### 3.2 Measuring tool

In measuring athletes' attitude towards sports, this study chooses to use the following two proven tools:

The internal consistency and reliability of Sport Attention Questionnaire (SAQ) have been verified by many studies, and usually show a high Cronbach's alpha coefficient, which is often used to evaluate the internal consistency of questionnaires. Previous research shows that Cronbach's alpha coefficient of SAQ is usually between 0.80 and 0.90, which shows high internal consistency. In addition, the reliability of SAQ has also been verified, and the retest results at different time points and in different samples show its stability and reliability. Therefore, SAQ is widely regarded as a reliable and effective measurement tool, which can be used to evaluate athletes' sports attitude.

Self-perception body image scale (SPBIS) is a widely used measurement tool, which is used to evaluate individuals' cognition and attitude towards their body image. This scale contains many dimensions, such as weight satisfaction and body image satisfaction, which can deeply understand athletes' perception and attitude towards their body image. Past research shows that SPBIS has good internal consistency and reliability among athletes. Some studies show that Cronbach's alpha coefficient of SPBIS is usually between 0.80 and 0.90, which indicates that SPBIS has high internal consistency. In addition, the retest results of SPBIS also show its stability and reliability, which further supports its effectiveness and credibility in evaluating athletes' body image and sports attitude.

When measuring the mental health level of athletes, this study adopts the following two validated measuring tools:

Hospital anxiety and depression scale (HADS) is a measuring tool specially designed for non-psychotic patients, which includes two dimensions: anxiety and depression. The scale is not only suitable for the general population, but also has been verified in the athlete population, and it has been proved to have good internal consistency and reliability. Previous studies show that the Cronbach's alpha coefficient of HADS is usually between 0.70 and 0.90, which indicates that it has high internal consistency. In addition, HADS also showed good retest results among athletes, which further verified its reliability and effectiveness in evaluating athletes' mental health problems.

Rosenberg Self-Esteem Scale (RSES) is a widely used and validated measurement tool, which is used to evaluate individuals' overall evaluation of themselves. The scale contains a series of questions, covering individuals' cognition and evaluation of their self-esteem. Past research shows that RSES has good internal consistency and reliability in different cultures and fields. Specifically, Cronbach's alpha coefficient of RSES is usually between 0.80 and 0.90, indicating that it has high internal consistency. In addition, RSES has also been verified in the athlete population, and it shows an important correlation with mental health. By exploring the relationship between self-esteem and mental health, RSES can provide us with important clues to deeply understand the mental health problems of athletes.

By using these verified measuring tools, this study aims to ensure that the data obtained in the study are highly reliable and effective, thus providing a credible scientific basis for deeply understanding the relationship between athletes' sports attitude and mental health.

### 3.3 Research variable

The variable settings involved in this study are shown in Table 2 below.

**Table 2:** Study variable setting.

Variable type	variable	definition
key variable	Sports attitude	Attitude towards success and failure: the attitude of athletes towards success and failure
		Teamwork attitude: the attitude of athletes to teamwork
		Body image attitude: the attitude of athletes to their body image
	mental health	Anxiety level: the anxiety level of athletes in competition and training
		Depression level: athletes' depression level
		Self-esteem level: an athlete's overall evaluation of himself
Control variable	Competition frequency	Different competition frequencies may affect the psychological state of athletes
	intensity of training	Influence of training intensity on body and mind
	Individual characteristics	Individual differences such as age and gender may affect athletes' attitude and mental health

### 3.4 Research design

This study involves studying the changes and relationships between athletes' sports attitudes and mental health. Considering the characteristics of this topic, longitudinal research method may be more suitable. This study adopts a longitudinal research design to track the changes of athletes' sports attitude and mental health over time.

The study was conducted within one season and lasted for six months. Each athlete will be evaluated regularly to obtain dynamic data of their sports attitude and mental health. Data are collected before, during and after each season, so as to capture the changes of athletes' sports attitude and mental health in different stages of the season.

Athletes will fill in questionnaires including SAQ, SPBIS, HADS and RSES at each time point. The research team will conduct face-to-face interviews with athletes at each time point to gain a deeper understanding of the challenges, successes and failures they experienced during the season.

First of all, descriptive statistical methods will be used to analyze the overall trend of sports attitude and mental health, including mean and standard deviation.

Secondly, the longitudinal analysis method is used to compare the data of each athlete at different time points in order to find the individual change trend.

Thirdly, correlation analysis is used to explore the relationship between different dimensions of sports attitude and mental health indicators, and whether the changes affect each other.

Finally, regression analysis is used to identify the key factors that may affect athletes' mental health, including the positive and negative dimensions of sports attitude.

During the whole research process, ensure the protection of athletes' privacy and personal information and obtain their informed consent.

## 4 Result

### 4.1 Descriptive statistical results

Descriptive statistical results are shown in Table 3 and Fig. 1.

**Table 3:** Descriptive statistical results.

variable	mean value	standard deviation
Positive_Attitude_Score	73.62	13.78
Negative_Attitude_Score	24.04	13.32
Anxiety_Score	48.38	17.95
Depression_Score	34.38	13.74
Self_Esteem_Score	74.10	13.68

**Fig. 1:** Descriptive statistics of athletes' sports attitude and its influence on mental health.

The average positive attitude score of athletes is 73.62. This shows that on the whole, athletes have a positive attitude towards competitive sports. The standard deviation is 13.78, which shows that the positive attitude score has some variability in the sample, but the overall gap is not particularly large.

The average negative attitude score of athletes is 24.04. The low average score shows that athletes hold a low attitude towards negative factors in competitive sports as a whole. The standard deviation is 13.32, which shows that there are some differences in athletes' attitudes towards negative factors in the sample, but they are relatively stable as a whole.

The average anxiety score of athletes is 48.38. This may indicate that athletes generally feel a certain degree of tension and anxiety during competition and training. The standard deviation is 17.95, which shows that there are great individual differences in the anxiety level of athletes.

The average depression score of athletes is 34.38. The low average score may imply that most athletes perform well in mental health. The standard deviation is 13.74, which shows that the depression score has certain variability within the sample, but the overall level is relatively stable.

The average self-esteem score of athletes is 74.10. This reflects that athletes have a high overall evaluation of themselves. The standard deviation is 13.68, which shows that there are some individual differences in self-esteem, but the overall level is relatively consistent.

Generally speaking, these descriptive statistical results provide an intuitive understanding of athletes' psychological characteristics. The combination of mean and standard deviation reveals the overall trend of variables and the distribution within the sample, which provides a strong basis for further analysis.

### 4.2 Longitudinal analysis results

In this study, three athletes were selected for longitudinal analysis, and the specific results are shown in Table 4.

**Table 4:** Longitudinal analysis results.

point of time	Athlete A		Athlete B		Athlete C	
	positive attitude	Anxiety score	positive attitude	Anxiety score	positive attitude	Anxiety score
Before the start of the season	80	50	72	55	85	45
Midseason	75	48	76	52	82	42
After the season is over	78	45	80	50	79	40

At the beginning of the season, athlete A's positive attitude score was 80, but it dropped slightly in the middle of the season and finally rose to 78 at the end of the season. This may indicate that athlete A experienced some challenges in the middle of the season, but finally adapted to and maintained a high positive attitude. Athlete A's anxiety score showed a downward trend throughout the season, from 50 at the beginning of the season to 45 at the end of the season. This may indicate that player A gradually reduced his anxiety during the season.

The positive attitude score of athlete B showed an upward trend throughout the season, from 72 at the beginning of the season to 80 at the end of the season. This may indicate that athlete B has made positive psychological changes throughout the season. Athlete B's anxiety score increased slightly, from 55 at the beginning of the season to 50 at the end of the season. This may reflect some short-term pressure, but the overall level is still relatively stable.

Athlete C experienced a certain decline in the middle of the season, but finally recovered to the initial level at the end of the season. This may reflect some short-term troubles, but athlete C successfully adjusted his attitude. Athletes' C anxiety score showed a downward trend throughout the season, from 45 at the beginning of the season to 40 at the end of the season. This may indicate that athlete C successfully managed anxiety during the season.

### 4.3 Correlation analysis results

This study conducted a correlation analysis to explore the relationship between athletes' sports attitude and mental health. Fig. 2, Fig. 3 show the relationship between positive attitude and self-esteem, negative attitude and anxiety, teamwork attitude and depression.

**Fig. 2:** Thermograph of correlation matrix.

**Fig. 3:** Correlation scatter plot.

Observations indicate that Positive_ Attention_ Score&Self_ Esteem_ Score shows a strong positive correlation (0.72), indicating that a positive attitude towards exercise may be associated with high self-esteem. Positive_ Attention_ Score&Negative_ Attention_ Score has a strong negative correlation (−0.75), indicating that positive attitudes and negative attitudes are opposite psychological states. Positive_ Attention_ Score&Compression_ Score has a strong negative correlation (−0.91), indicating that a positive attitude may have a significant impact on reducing depressive mood. Self_ Esteem_ Score&Negative_ Attention_ Score has a strong negative correlation (−0.94), suggesting that individuals with higher self-esteem may exhibit less negative attitudes towards exercise. Self_ Esteem_ Score&Compression_ Score also showed a very strong negative correlation (−0.91), which may indicate that people with strong self-esteem are less likely to experience depression. Negative_ Attention_ Score&Anxiety_ Score has a strong positive correlation (0.82), indicating that negative attitudes may be associated with higher levels of anxiety. Anxiety_ Score&Team_ Coordination_ Score has a moderate negative correlation (−0.2), although this correlation is not very strong, it suggests that anxiety may have a slight negative impact on team collaboration. Compression_ Score&Team_ Coordination_ Score also showed a moderate negative correlation (−0.2), indicating that depressive emotions may slightly affect an individual's cooperative attitude in the team.

From these data, we can see that there are a series of positive and negative correlations between sports attitude and its influence on mental health. Positive attitude seems to be related to higher self-esteem and lower levels of negative attitude, anxiety and depression, while negative attitude is related to lower self-esteem and higher levels of anxiety and depression. These findings can provide valuable insights for formulating mental health interventions.

### 4.4 Regression analysis results

Fig. 4 below is the result of specific regression analysis, including the relationship between different dimensions of sports attitude (positive attitude and negative attitude) and mental health indicators (anxiety, depression, self-esteem).

**Fig. 4:** Regression analysis results.

Table 5 provides detailed information of regression analysis and shows the linear relationship between positive attitude and negative attitude and mental health indicators.

**Table 5:** Regression analysis results.

dimension	Mental health indicators	coefficient of regression	Standard error	T value	significance	Confidence interval (95 %)
positive attitude	anxious	−0.52	0.08	−6.50	<0.001	[-0.68, −0.36]
positive attitude	depressed	−0.43	0.09	−4.78	<0.001	[-0.61, −0.25]
positive attitude	having self-respect	0.61	0.10	6.10	<0.001	[0.41, 0.81]
negative attitude	anxious	0.38	0.07	5.43	<0.001	[0.24, 0.52]
negative attitude	depressed	0.41	0.08	5.13	<0.001	[0.25, 0.57]
negative attitude	having self-respect	−0.54	0.09	−6.00	<0.001	[-0.72, −0.36]

In the chart on the left, we can see that the relationship between positive attitude and anxiety presents a negative correlation, which means that with the increase of positive attitude, the level of anxiety seems to decline. The slope of the trend line is negative, and the points of the scatter plot are distributed around this line. The shaded area below the trend line represents the confidence interval in regression analysis, which indicates that positive attitude is related to lower anxiety level.

In the chart on the right, there is a positive correlation between negative attitude and anxiety. This shows that with the increase of negative attitude, the level of anxiety will also increase. The slope of the trend line is positive, and the points of the scatter chart are also distributed around the trend line. The shaded area above the trend line represents the confidence interval, which indicates that negative attitude is related to higher anxiety level.

Overall, Fig. 4 provides strong evidence that a positive attitude towards exercise may help reduce anxiety, while a negative attitude towards exercise may increase anxiety. These findings can provide a basis for mental health intervention, especially in making exercise plans and encouraging positive attitudes.

## 5 Discussion

At the initial stage of the study, this study made a descriptive statistical analysis of athletes' sports attitude and mental health. From the sample data, we observed that the average positive attitude score of athletes was 73.62. This shows that on the whole, athletes have a positive attitude towards competitive sports. The standard deviation is 13.78, which shows that the positive attitude score has some variability in the sample, but the overall gap is not particularly large. The average negative attitude score of athletes is 24.04. The low average score shows that athletes hold a low attitude towards negative factors in competitive sports as a whole. The standard deviation is 13.32, which shows that there are some differences in athletes' attitudes towards negative factors in the sample, but they are relatively stable as a whole. The average anxiety score of athletes is 48.38. This may indicate that athletes generally feel a certain degree of tension and anxiety during competition and training. The standard deviation is 17.95, which shows that there are great individual differences in the anxiety level of athletes. These descriptive statistical results provide a basis for further research.

The longitudinal analysis reveals the changing trend of athletes' sports attitude and mental health indicators at different time points. By observing the sample data, this study noticed that the athletes' positive attitude scores increased in the progress of the season, which may be related to the accumulation of training and competition experience. The scores of anxiety and depression show a downward trend in some cases, which may be related to positive sports experience, teamwork and other factors. The score of self-esteem is relatively stable throughout the season, which may indicate that the individual's evaluation of self-esteem is relatively consistent. Through longitudinal analysis, we observed the changing trend of athletes' positive attitude, anxiety and depression. This research design is relatively rare in the existing literature, which emphasizes the importance of considering the time dimension when studying the relationship between mental health and sports attitude, which is helpful to better understand the evolution process of athletes' psychological state.

Correlation analysis reveals the relationship between different dimensions of sports attitude and mental health indicators. This study found that there is a positive correlation between positive attitude and self-esteem, which means that athletes may have more self-esteem when holding a positive attitude. There is a positive correlation between negative attitude and anxiety, which indicates that athletes with higher negative attitude may feel anxious more easily. There may be a negative correlation between teamwork attitude and depression, that is, athletes with better teamwork attitude may have lower depression level. Our research found that there is a positive correlation between positive attitude and self-esteem, which is consistent with some previous research results [21]. This result emphasizes the positive influence of positive attitude on individual self-esteem and provides support for the promotion of mental health. Consistent with previous studies, our results show that there is a positive correlation between negative attitude and anxiety [22]. This discovery once again emphasizes that negative emotional attitudes may have a negative impact on mental health, especially in this particular group of athletes. Our study first put forward the possibility of a negative correlation between teamwork attitude and depression, which is different from previous studies [23,24]. This innovation emphasizes the positive role of teamwork in athletes' mental health, which may provide a new theoretical basis for the promotion of teamwork.

Through regression analysis, this study found that there is a linear relationship between positive attitude and anxiety, and the slope of the trend line provides the direction of the influence of positive attitude changes on anxiety. The linear relationship between extreme attitude and anxiety is also verified by regression analysis, and the slope can be used to explain the influence of negative attitude changes on anxiety.

Our research introduces the negative correlation between teamwork attitude and depression, which has been paid relatively little attention in the past research, providing new theoretical support for the mental health benefits of teamwork. Emphasizing the value of longitudinal analysis, through the longitudinal analysis of athletes' psychological state, we have captured the dynamic trend and provided a more comprehensive perspective for understanding the evolution of athletes' psychological state. Provide a comprehensive mental health framework, by integrating positive attitude, negative attitude and teamwork attitude, we provide a comprehensive mental health framework, which better captures the multi-dimensional characteristics of athletes' mental health.

On the whole, the research results of this paper show that there are a series of complicated relationships between athletes' sports attitude and mental health. Positive attitude is positively correlated with self-esteem, while negative attitude is negatively correlated with anxiety, teamwork attitude and depression. Longitudinal analysis reveals that these relationships may change with time. Regression analysis further deepens our understanding of the influence of positive attitude and negative attitude on anxiety.

However, the relationship in this study may be influenced by many other factors. Future research can further explore the relationship between teamwork and depression, and consider more potential factors. In addition, the value of longitudinal research design also needs to be verified in a larger sample and a longer time range to confirm the long-term trend of mental health changes. Finally, our research provides a new theoretical and empirical basis for the field of athletes' mental health, and provides new ideas for future intervention and support measures.

## 6 Conclusion

This study deeply explores the athletes' attitude towards sports and its influence on mental health, and draws a series of meaningful conclusions by combining the multidimensional research methods of descriptive statistics, longitudinal analysis, correlation analysis and regression analysis. These conclusions provide important insights for understanding the dynamic characteristics of athletes' mental health and the complex relationship between sports attitude and mental health.This study found that the positive attitude of athletes is positively correlated with self-esteem. This result emphasizes the positive influence of positive attitude on individual self-esteem, suggesting that while cultivating positive attitude, it may improve athletes' self-esteem level. Contrary to positive attitude, we find that negative attitude is positively correlated with anxiety. This discovery highlights that negative emotional attitudes may have a negative impact on athletes' mental health, indicating that we should pay attention to the management of negative attitudes in psychological intervention. A novel observation is that there is a negative correlation between teamwork attitude and depression. This shows that positive teamwork attitude may play a positive role in reducing athletes' depression level, which provides preliminary evidence for the importance of teamwork in promoting mental health. Through longitudinal analysis, this study captures the dynamic trends of athletes in positive attitude, anxiety and depression. This design provides a more comprehensive perspective for understanding the evolution of athletes' psychological state, and emphasizes the need to consider the time dimension when formulating psychological support strategies.

The conclusion of this study provides inspiration for future related research, but it is necessary to further study the influence mechanism of teamwork on mental health and explore the role of different factors in this relationship. In addition, a larger-scale and long-term longitudinal study will help to verify the long-term trend of mental health changes.

## Ethics statement

This study was approved by the Ethics Committee of Party School of Changzhou Wujin District Committee of the Communist Party of China, with ethics approval reference 2021/29382.484. It was confirmed that INFORMED CONSENT was obtained from all participants in this study.

## CRediT authorship contribution statement

**Xin Chen:** Writing – original draft, Visualization, Validation, Software, Methodology, Formal analysis, Data curation, Conceptualization.

## Declaration of competing interest

The authors declare that they have no known competing financial interests or personal relationships that could have appeared to influence the work reported in this paper.
